# Automatic Segmentation of Left Ventricle in Echocardiography Based on YOLOv3 Model to Achieve Constraint and Positioning

**DOI:** 10.1155/2021/3772129

**Published:** 2021-05-16

**Authors:** Zhemin Zhuang, Pengcheng Jin, Alex Noel Joseph Raj, Ye Yuan, Shuxin Zhuang

**Affiliations:** ^1^Department of Electronic Engineering, Shantou University, Shantou 515063, China; ^2^Guangdong Provincial Key Laboratory of Digital Signal and Image Processing, Shantou University, Shantou 515063, China

## Abstract

Cardiovascular disease (CVD) is the most common type of disease and has a high fatality rate in humans. Early diagnosis is critical for the prognosis of CVD. Before using myocardial tissue strain, strain rate, and other indicators to evaluate and analyze cardiac function, accurate segmentation of the left ventricle (LV) endocardium is vital for ensuring the accuracy of subsequent diagnosis. For accurate segmentation of the LV endocardium, this paper proposes the extraction of the LV region features based on the YOLOv3 model to locate the positions of the apex and bottom of the LV, as well as that of the LV region; thereafter, the subimages of the LV can be obtained, and based on the Markov random field (MRF) model, preliminary identification and binarization of the myocardium of the LV subimages can be realized. Finally, under the constraints of the three aforementioned positions of the LV, precise segmentation and extraction of the LV endocardium can be achieved using nonlinear least-squares curve fitting and edge approximation. The experiments show that the proposed segmentation evaluation indices of the method, including computation speed (fps), Dice, mean absolute distance (MAD), and Hausdorff distance (HD), can reach 2.1–2.25 fps, 93.57 ± 1.97%, 2.57 ± 0.89 mm, and 6.68 ± 1.78 mm, respectively. This indicates that the suggested method has better segmentation accuracy and robustness than existing techniques.

## 1. Introduction

Cardiovascular diseases (CVDs) are one of the most common diseases affecting humans. “Global Burden of Cardiovascular Diseases and Risk Factors, 1990–2019,” published in [1], shows that the incidence and mortality of CVD worldwide have been increasing since 1990 and that the mortality of CVD ranks first and is far higher than that of other diseases. Therefore, early detection and diagnosis of cardiac disease through various means is crucial for reducing the prevalence and mortality of CVD and improving the quality of life of patients [2].

Compared with X-ray coronary angiography, myocardial contrast echocardiography, computed tomography, and magnetic resonance imaging, the use of ultrasound for the screening and diagnosis of heart function and disease has great advantages. Using an ultrasound instrument, the heart and blood vessels, the movement of the ventricular wall, and the opening and closing of the valve can be observed dynamically in real time through flexible operation from multiple directions and angles. In addition, ultrasound has many advantages, such as safety and noninvasiveness, high diagnostic accuracy, and rapid inspection, and has become one of the most used and important examination methods for heart disease.

At present, the diagnosis of heart diseases based on ultrasound technology usually focuses on the analysis of the left ventricle (LV). The LV is responsible for blood supply to the body. Based on the changes in the LV, indicators such as LV end-diastolic volume, LV end-systolic volume, LV ejection fraction (EF), and LV stroke volume can be obtained. To obtain the indicators above, accurate positioning and segmentation of the LV on echocardiography are very important.

Clinically, the segmentation methods for LV ultrasound images can be classified into manual and automatic methods. The manual segmentation method requires the user to outline the region of interest manually. Marking the position or contour of the LV manually is tedious and time-consuming, and there are subjective differences among different observers. The automatic segmentation method is superior to the manual segmentation method [3, 4]. Usually, the automatic segmentation method of LV ultrasound images includes two steps.

First, it is necessary to determine the position of the LV in the ultrasound images. Methods such as scale-invariant feature transformation [5] and histogram of oriented gradient [6] can be used to determine the position of the LV. However, the shape and appearance of the LV corresponding to different individuals are usually different, so these methods cannot accurately identify the position of the LV, and the segmentation accuracy of LV is also affected. Recently, the application of deep learning models for target detection and localization has attracted increasing attention [7, 8]. Compared with the faster R-CNN model [9] and the single-shot multibox detector model [10], the YOLOv3 model [11] has a higher detection speed and accuracy. Therefore, a method based on the YOLOv3 model is proposed herein for accurate positioning and segmentation of the LV.

Second, after the LV in the ultrasound image is accurately located, the LV can be segmented. Methods such as structured random forest based on machine learning [12] have been proposed for LV segmentation; however, such methods require manual selection of space features. Dong et al. [13] developed a deep fusion network and deformable model to achieve LV segmentation in 3-D echocardiography. Smistad et al. [14] successfully segmented the LV in two-dimensional ultrasound images based on the U-Net method. Oktay et al. [15] further extended the U-Net model to improve the accuracy of LV segmentation. However, these methods usually require significant morphological features or prior knowledge and have the disadvantages of poor real-time performance and high computing power requirements. Traditional image processing methods, such as a motion-based method (Kalman filter) [16], deformable models (BEAS, level-set) [17, 18], graph-based approach (graphcut) [19], active appearance model [20], and atlas-based method [21], have been proven to have high segmentation speed and robustness in heart image segmentation. Therefore, the YOLOv3 model and the traditional statistical shape model are combined in this study to achieve fast and accurate LV segmentation in ultrasound images.

Herein, an automatic segmentation method based on the YOLOv3 model to satisfy the relevant constraints and achieve appropriate positioning is proposed for accurate segmentation of the LV endocardium. The results of experiments conducted using the proposed method show that the segmentation evaluation indices, including the computation speed (fps), Dice, mean absolute distance (MAD), and Hausdorff distance (HD), can reach 2.1–2.25 fps, 93.57 ± 1.97%, 2.57 ± 0.89 mm, and 6.68 ± 1.78 mm, respectively.

## 2. Method

To obtain clinical indicators such as EF, strain, and strain rate of the LV on echocardiography, accurate segmentation of the LV is crucial. In this study, the YOLOv3 model is first used to determine the three positions of the apex and bottom of the LV, as well as the location of the LV region. Then, based on the Markov random field (MRF) model with the iterated conditional mode (ICM), preliminary identification and binarization of the myocardium of the LV subimages are performed, and under the three constraint points of the LV, the left and right parts of the myocardium in the LV subimages are located. Finally, when approaching the edge of the myocardium, the B-spline method is used to smooth the edge of the endocardium, and then, accurate segmentation and extraction of the LV endocardium are achieved. Speckle noise and artifacts in ultrasound images can lead to the loss of borders and edges during image segmentation; therefore, when approaching the LV endocardium, a morphological mask is applied to eliminate the interference from speckle noise and edge artifacts inside the LV cavity.  Figure 1 presents the block diagram of the proposed technique.

## 3. Segmentation of LV Endocardium Based on YOLOv3 for Positioning and Restraint

### 3.1. LV Localization and Collection of Restraint Points Based on the YOLOv3 Model

There are large differences in the shape of the LV in different echocardiogram frames. In addition, due to the interference of the mitral valve, as well as the influence of noise, artifacts, and frame-to-frame drift, traditional methods cannot locate the LV position well or extract the endocardium accurately. Therefore, this study proposes to use the target detection model YOLOv3 to realize the positioning of the LV region and the three ventricular constraint points in echocardiography. From Figure 2, the YOLOv3 model consists of the following: a general feature extraction network based on the Darknet-53 network, a multibranch deep feature extraction network, and a multiscale target area bounding box detection network.

In Figure 2, for the general feature extraction network, the convolutional network (Conv), batch normalization (BN) layer, and linear activation function (Leaky ReLU) constitute Darknetconv2d BN Leaky (DBL), which extracts the general features of cardiac ultrasound images. The DBL is also the basic block of deep feature extraction networks. Concurrently, to solve problems such as the disappearance of gradients due to the deep network structure, DarkNet53 uses the jump structure to form Res_unit, Resblock_body, and Res_Module in multiple DBLs.

For the deep-level feature extraction network, YOLOv3 forms a multibranch network and a Concat layer through the route structure. Simultaneously, YOLOv3 uses a bilinear upsampling layer to expand the feature map to form three branch networks for locating target areas of three different scales; through these three branch networks, the feature matrix of the LV ultrasound image can be obtained. In practice, it is difficult to obtain enough labeled LV images, and to avoid overfitting, transfer learning is applied in this study to train the entire feature extraction network: first, load the weight parameters obtained based on the VOC dataset [22] and then fine-tune the weight parameters of the feature extraction network using the labeled heart dataset.

After the feature matrices of the LV ultrasound images of the heart are obtained, they are input into the detection network to obtain the positioning matrices. The YOLOv3 model divides the original input images into three types of *S* × *S* grids (i.e., 13 × 13, 26 × 26, and 52 × 52) for positioning the target area; hence, three types of positioning matrices with different dimensions are obtained. As shown in Figure 2, the *y*_1_ matrix corresponding to a 13 × 13 grid is used to detect a large target area and is used to locate the LV area in this study; the *y*_2_ and *y*_3_ matrices correspond to the 26 × 26 and 52 × 52 grids, respectively, which are used to locate three ventricular restraint points in this study.

Each grid corresponds to a (*B* + *O*) × anchors-dimensional positioning vector, where *B* is the bounding box of the target area, composed of (*b*_*x*_, *b*_*y*_, *b*_*w*_, *b*_*h*_, *b*_*c*_), corresponding to the center abscissa, ordinate, width, height, and confidence from the center of the target area, respectively, and *O* is the number of types of the target area. In this study, there are four types of targets: the LV region and three ventricular constraint points. anchors are the number of anchor frames in the positioning matrix; the number of anchor frames with three scales in this study is three.

The anchor box is used to describe the length and width of the target area in this study, and the relationship between the anchor box and bounding box is shown in Equation (1).

(1) $$\begin{array}{c} \begin{array}{c} b_{x}=\sigma \left(t_{x}\right)+C_{x},\\ b_{y}=\sigma \left(t_{y}\right)+C_{y},\\ \begin{array}{c} b_{w}=P_{w}e^{t_{w}},\\ b_{h}=P_{h}e^{t_{h}}, \end{array} \end{array} \end{array}$$

where *C*_*x*_, *C*_*y*_, *P*_*w*_, and *P*_*h*_ are the abscissa, ordinate, and the width and height of the upper left corner of the grid where the center point of the anchor frame is located, respectively; *σ*(∙) is the sigmoid activation function; *t*_*x*_ and *t*_*y*_ are the abscissa and ordinate offsets of the center of the anchor frame; and *t*_*w*_ and *t*_*h*_ are the changes in the length and width of the anchor frame.

In this study, the target area in the training set is divided into nine anchor boxes using the *K*-means [23] clustering algorithm, and each anchor box is represented as (*w*, *h*). For these anchor boxes, three small anchor boxes ((0 × 0), (11 × 13), and (11 × 15)) (i.e., the *y*_1_ matrix in Figure 2) are used to locate the LV area: three medium anchor boxes ((13 × 15), (14 × 20), and (15 × 17)), and three large anchor boxes ((16 × 22), (110 × 218), and (146 × 323)) (i.e., the *y*_2_ and *y*_3_ matrices in Figure 2) are used for the positioning of three constraint points.

### 3.2. Extraction of Endocardium Based on Constraint Points

The three positions of the apex and bottom of the LV, as well as the positioning of the LV area, can be found by the YOLOv3 model mentioned above. Then, based on the MRF model, the binarization and preliminary identification of the LV myocardial region in the subimages can be performed. Under the constraints of the three position points of the apex and bottom of the LV, curve fitting was performed on the left and right myocardial parts in the LV subimages, and the edge of the endocardium was approximated to realize accurate segmentation of the LV endocardium, and the B-spline method was also employed to smooth the edge of the LV endocardium.

#### 3.2.1. Binarization of LV Myocardium Based on MRF Model

Before the LV myocardial images are binarized, to reduce the influence of speckle and noise in echocardiograms, the echocardiograms are denoised on the premise of preserving the characteristics of the LV myocardium. First, the LV subimages are smoothed via 2-D adaptive Wiener noise-removal filtering [24], the local neighborhood size is set to (5 × 5), and then, the pixel-wise Wiener filter can be constructed using Equation (2).

(2) $$\begin{array}{c} b\left(n_{1},n_{2}\right)=\mu +\frac{\sigma^{2}-\nu^{2}}{\sigma^{2}}\left(a\left(n_{1},n_{2}\right)-\mu \right), \end{array}$$

where *μ* and *σ*^2^ are the local mean and variance around each pixel, respectively, and *ν*^2^ is the variance of the noise. The Wiener filter adjusts itself to the local image variance, i.e., when the variance is large, a minor smoothing operation is performed by the Wiener filter whereas when variance is small, the Wiener filter performs a major smoothing.

The MRF model utilizes the correlation between the upper and lower adjacent pixels in the image; thus, the spatial connectivity and edge smoothness of the binarized region can be improved. Therefore, an MRF model based on the ICM algorithm was used in this study to binarize and initially identify the myocardial region.

Assume that *X* and *Y* are random fields on a two-dimensional plane, where *X* = {*x*_*i*_, *i* = 1, 2, 3, ⋯, *M* × *N*} represents the input image and *Y* = {*y*_*i*_, *i* = 1, 2, 3, ⋯, *M* × *N*} represents the labeling field, where *M* and *N* represent the rows and columns of the image, respectively. In this study, the *K*-means clustering method was used to obtain the initial marker field, and the category was set to 2.

Considering the input images as an MRF model, the image segmentation problem can be transformed into an optimization problem using the ICM algorithm. According to the Bayesian principle, the posterior probability distribution of MRF is as follows:

(3) $$\begin{array}{c} P\left(X=x\;|\;Y=y\right)=\frac{P\left(Y=y\;|\;X=x\right)P\left(X=x\right)}{P\left(Y=y\right)}, \end{array}$$

where *P*(*Y* = *y*) is a constant for a given LV subimage, *P*(*X* = *x*) is the prior probability of the label domain, and *P*(*Y* = *y* | *X* = *x*) is the likelihood function.

When binarizing the LV images, the optimal labels can be obtained by maximizing the posterior probability of Equation (3).

(4) $$\begin{array}{c} P{\left(X=x\;|\;Y=y\right)}_{MAP}=\text{argmax}\left\{P\left(Y=y\;|\;X=x\right)P\left(X=x\right)\right\}. \end{array}$$

The prior probability *P*(*X* = *x*) in the MRF neighborhood system can be expressed using the Gibbs distribution function [25]. Then, based on the Gibbs distribution, the prior probability *P*(*X* = *x*) of the marker field can be characterized as follows:

(5) $$\begin{array}{c} P\left(X=x\right)=\frac{1}{Z}\exp\left[-\frac{E\left(x\right)}{T}\right], \end{array}$$

where *Z* = ∑_*x*∈*Ω*_exp[−*E*(*x*)/*T*] is a normalized constant, *E*(*x*) = ∑_*c*∈*S*_*V*_*c*_(*x*) is the energy function, *V*_*c*_(*x*) is the potential function, and *T* is the temperature parameter, which is usually set to 1 [26].

Similarly, the posterior probability *P*(*X* = *x* | *Y* = *y*) can also be expressed by an energy function, as shown in Equation (6).

(6) $$\begin{array}{c} P\left(X=x\;|\;Y=y\right)=\frac{1}{Z}\exp\left[-\frac{E\left(x\;|\;y\right)}{T}\right]. \end{array}$$

Substituting Equations (5) and (6) into Equation (4), and taking the logarithms on both sides of the equation simultaneously, the product form is transformed into a summation form, and the result is as follows:

(7) $$\begin{array}{c} E\left(x\;|\;y\right)=\text{argmax}\left\{E\left(y\;|\;x\right)+E\left(x\right)\right\}, \end{array}$$

where *E*(*x* | *y*) represents the minimized energy function, *E*(*y* | *x*) is the likelihood function energy of pixel *x*, and *E*(*x*) is the prior probability energy corresponding to pixel *x*. Therefore, the final energy relationship can be expressed as Equation (8).

(8) $$\begin{array}{c} E\left(x_{F}\;|\;y\right)=E\left(y\;|\;x\right)+E\left(x\right), \end{array}$$

where *x*_*F*_ is the final segmentation mark.

The ICM algorithm is used to optimize Equation (8), i.e., to minimize the energy function *E*(*x*_*F*_ | *y*). Finally, the binarization results of LV myocardium images can be obtained and are shown in Figure 3. As shown in Figure 3, the LV myocardium can be clearly observed after the original LV images are binarized using the MRF model.

#### 3.2.2. Segmentation and Extraction of LV Myocardium Based on Position Constraints

After binarizing the original LV images based on the MRF model, the positioning curve of the LV myocardium will be fitted based on the position constraints. Firstly, divide the LV into the left and right regions and then use the nonlinear least squares (NLS) method to perform curve fitting on the two regions. Because only the LV endocardium is approximated in this study, three constraint points are used to limit and constrain the fitted curve.

In this study, a polynomial model based on the NLS method is employed to fit the left and right segments, respectively, as shown in Equation (9).

(9) $$\begin{array}{c} F\left(x\right)=a_{1}x^{m}+a_{2}x^{m-1}+\cdots +a_{m}x+a_{m+1}, \end{array}$$

where *a*_1_, *a*_2_, ⋯, *a*_*m*+1_ represents the fitting coefficient of the polynomial, and *m* is the polynomial degree; in this study, the polynomial degree *m* is set to 3.

For a given set of coordinate points {(*x*_*i*_, *y*_*i*_): *i* = 1, 2, ⋯, *n*}, the polynomial fitting error equation can be written as Equation (10).

(10) $$\begin{array}{c} V=BX-L, \end{array}$$

where

(11) $$\begin{array}{c} B=\left(\begin{array}{c} x_{1}^{m}\\ x_{2}^{m}\\ \vdots \\ x_{n}^{m} \end{array}\begin{array}{c} x_{1}^{m-1}\\ x_{2}^{m-1}\\ \vdots \\ x_{n}^{m-1} \end{array}\begin{array}{c} \cdots \\ \cdots \\ \vdots \\ \cdots \end{array}\begin{array}{c} x_{1}\\ x_{2}\\ \vdots \\ x_{n} \end{array}\right),\\ X=\left(\begin{array}{c} a_{1}\\ a_{2}\\ \vdots \\ a_{m+1} \end{array}\right),\\ L=\left(\begin{array}{c} F\left(x_{1}\right)\\ F\left(x_{2}\right)\\ \vdots \\ F\left(x_{n}\right) \end{array}\right). \end{array}$$

Based on the NLS method, the estimated value of *X* can be obtained as follows:

(12) $$\begin{array}{c} X={\left(B^{T}B\right)}^{-1}B^{T}L. \end{array}$$

Substituting the result obtained from Equation (12) into Equation (9), the LV myocardial positioning fitting curve can be obtained, as shown in Figure 4, where the red boxes in Figure 4(a) are the constraint points obtained by the YOLOv3 model. The obtained three constraint points are used for the constraint of the myocardial fitting curve.  Figure 4(b) is the positioning fitting curve without restraint, and Figure 4(c) is the constrained positioning fitting curve.

As shown in Figure 4, under the three constraint points obtained based on the YOLOv3 model, the positioning curve of the myocardium can be accurately determined in the LV.

To mitigate the influence of speckle noise around the LV myocardium, the binary LV images obtained based on the MRF model are processed using the morphological masking method. After the initial positioning of the LV myocardium is achieved, the endocardium is approached based on the three constraint points, the edge of the endocardium is smoothed by the B-spline method [27], and the segmentation and extraction of the LV endocardium can be realized as shown in Figure 5.

## 4. Results

The cardiac ultrasound imaging data used in this study were provided by the Ultrasound Imaging Department of the First Affiliated Hospital of Medical College of Shantou University.

### 4.1. Evaluation Criteria

For target detection tasks, the average precision (AP) indicator [28] is commonly used to evaluate whether a model can detect a target class accurately. The AP is computed as the intersection of union (IOU) between the detection bounding box and the label bounding box. When the IOU of the detection bounding box and the label bounding box is greater than the set IOU threshold, it is considered that the model detects the target correctly. Subsequently, the AP value of the target class is calculated. In practice, the IOU threshold is usually set to 0.5, and the corresponding AP indicator is called AP50. For a model used to detect multiple target classes, the mean average precision (mAP) can comprehensively evaluate the performance of the model, i.e., compute the average value of the AP values of all target classes.

A precision-recall (*P*‐*R*) curve [29] is shown with precision and recall as the vertical and horizontal axis, respectively. Also the size of the area under the *P*‐*R* curve can comprehensively reflect the performance of a model for detecting the target.

AP can be expressed as

(13) $$\begin{array}{c} \text{AP}=\int_{0}^{1}P\left(R\right)dR, \end{array}$$

where *P* and *R* represents the precision and recall rates, respectively. The precision and recall in the *P*‐*R* curve are calculated using Equations (14) and (15), respectively.

(14) $$\begin{array}{c} \text{precision}=\frac{\text{TP}}{\text{TP}+\text{FP}}, \end{array}$$

(15) $$\begin{array}{c} \text{recall}=\frac{\text{TP}}{\text{TP}+\text{FN}}, \end{array}$$

where TP, FP, and FN represent the true positive, the false positive and the false negative, respectively.

The Dice coefficient [30], MAD [31], and HD [32] parameters are used to evaluate the segmentation results of the LV endocardium:

(16) $$\begin{array}{c} \text{Dice}\left(S,G\right)=\frac{2\text{Area}\left(S\cap G\right)}{\text{Area}\left(S\right)+\text{Area}\left(G\right)},\\ \text{MAD}\left(A,B\right)=\frac{1}{2}\left\{\frac{1}{m}\overset{m}{\underset{i=1}{\sum }}d\left(a_{i},B\right)+\frac{1}{n}\overset{n}{\underset{j=1}{\sum }}d\left(b_{i},A\right)\right\},\\ \text{HD}\left(A,B\right)=\max\left\{\underset{i}{\max}\left\{d\left(a_{i},B\right)\right\},\underset{j}{\max}\left\{d\left(b_{j},A\right)\right\}\right\}, \end{array}$$

where *S* represents the myocardial area data obtained by different binarization methods, *G* is the gold standard data of the myocardial area, *A* = {*a*_1_, *a*_2_, ⋯, *a*_*m*_} is the endomyocardial edge data obtained by the method proposed in this paper, and *B* = {*b*_1_, *b*_2_, ⋯, *b*_*n*_} is the gold standard endomyocardial edge data.

### 4.2. LV and Restraint Point Positioning Model Based on YOLOv3

Table 1 illustrates the performance of the YOLOv3-based LV and bounding box positioning model on the test dataset using AP50. From Table 1, all the AP50 values of the four target regions formed by the LV and the three bounding boxes are above 92%, and the mAP value reaches 95.57%, which indicates that the model designed in this study can detect the LV and the three bounding box areas well and meet the requirements of LV myocardium segmentation.

The *P*‐*R* curve, which can intuitively evaluate whether the model can detect a target class well, is drawn based on the precision-recall value pairs calculated from different confidence values when the model detects a target class. The value of the area enclosed by the *P*‐*R* curve is the AP value.

The *P*‐*R* curve of the model on the test dataset is shown in Figure 6. It can also be seen from Figure 6 that the area under the four *P*‐*R* curves is sufficiently large, which indicates that the performance of the model is satisfactory.

### 4.3. LV Binarization

To analyze the effect of the MRF model on the binarization of the ultrasound LV images, the proposed method, traditional Otsu method, and *K*-means clustering algorithms were used to binarize the same LV image for comparison; the binarization results obtained by different methods were also compared with the gold standard, and the results are shown in Figure 7.

From Figure 7, it can be verified that the myocardial area obtained using the proposed model is closest to the gold standard.

For quantitative analysis, the Dice index is used for evaluation. The LV myocardial regions obtained by the Otsu method, *K*-means clustering algorithm, and the method based on MRF proposed in this paper are compared with the gold standard myocardial region obtained by manual segmentation by senior clinicians, and the corresponding Dice indices are obtained, and the results are shown in Table 2.

It can be seen from Table 2 that the Dice value corresponding to the proposed binarization method based on the MRF model is 0.88 ± 0.03, which is far greater than the Dice values corresponding to the Otsu method and *K*-means clustering algorithm, namely, the performance of the binarization method based on the MRF model proposed in this paper is much better than the other two methods. Therefore, the binarization method proposed in this study can fully meet the requirements for extraction of the LV myocardial region.

### 4.4. LV Endocardium Segmentation

In order to evaluate the performance of the method proposed in this paper, the same LV ultrasound images were segmented using different methods (listed in Table 3) along with the proposed method, and the segmentation results by different methods were compared with the gold standard obtained by manual segmentation by cardiologists, and five evaluation indicators including training set size, computation speed, Dice coefficient, MAD, and HD were used to evaluate the segmentation results. The results are shown in Table 3.

It can be seen from Table 3 that the proposed segmentation technique is superior to other methods in terms of various evaluation indicators. In particular, for the computation speed index, the method proposed in this paper has a great advantage, and owing to the use of transfer learning, the method uses less training data to obtain a better segmentation effect.

## 5. Discussion

In this paper, an automatic LV segmentation method based on the YOLOv3 model is proposed to determine the constraints and positioning. Through the YOLOv3 model, the three positions of the apex and bottom of the LV and LV area are positioned, and based on the MRF model, the LV myocardium subimages are binarized; under the limitation of the three constraint points of the LV, combined with NLS curve fitting and B-spline smoothing, the accurate segmentation and extraction of the LV can be realized. Experiments show that the suggested method can accurately and automatically identify and segment the LV in cardiac ultrasound images.

In the experimental section, a comparison is presented with other segmentation models. Hansson et al. [33] proposed an unsupervised segmentation method based on a Bayesian probability map. Although MADs corresponding to the aforementioned method and the method proposed herein are similar (which means that the two methods are similar in terms of segmentation accuracy), the computation speed of the latter is much higher than that of the former (see the computation speed indicator). The level set segmentation method proposed by Qin et al. [34] is unsupervised, does not require a training dataset, and can yield accurate segmentation results. However, owing to the need for sparse matrix transformation to identify the right ventricle, this method requires many training sets and a large processing time; in addition, it is necessary to readjust the parameters according to the movement of the heart, which will lead to unstable results. Compared with that of the aforementioned method, the MAD of the method proposed herein this paper is slightly lower, but the Dice value is better. In fact, the method proposed by Qin et al. is similar to our method in terms of segmentation accuracy. However, the method proposed herein is far superior in terms of the computation speed indicator. The method proposed by Carneiro and Nascimento [35] uses a deep neural network method to segment the systolic and end-diastolic contours and achieves high segmentation accuracy; however, a large number of datasets is required, and thus, a set of 496 images had to be established. Compared with this method, the method proposed herein only requires a small amount of data (252 frames) to obtain a suitable positioning effect; in terms of calculation speed, the method proposed herein this paper is significantly better than that proposed by Carneiro and Nascimento (see the corresponding computation speed index in Table 3). Finally, according to the computation speed, Dice, MAD, and HD, the automatic LV segmentation method based on constraints and positioning are better in the proposed technique than unconstrained positioning segmentation methods in terms of segmentation accuracy and computation speed.

In summary, if the segmentation accuracy indices (i.e., Dice, MAD, and HD) are considered, the method proposed is not the best, but it can be said that the method proposed in this paper is one of the best methods in terms of segmentation accuracy; however, if the computation speed, data volume, and segmentation accuracy are considered comprehensively, it can be said that the method proposed in this paper is the best. Compared with other methods, the proposed segmentation technique has significant advantages in terms of computation speed and the amount of data required. The method proposed in this study uses fewer data to obtain a good segmentation effect. It is well known that it is very difficult to obtain medical data in practice, thus obtaining a good segmentation effect based on a small amount of data is conducive to the clinical application of the algorithm. The computation speed is another important factor that affects the application of algorithms in clinical practice, and the algorithm proposed has significant advantages in terms of computation speed over the other methods.

## 6. Conclusions

Here, an automatic LV segmentation method based on the YOLOv3 model for constraint and positioning determination is proposed. Through the YOLOv3 model, the three positions of the apex and bottom of the LV and LV area are positioned, and based on the MRF model, the LV myocardium subimages are binarized; under the limitation of the three constraint points of the LV, combined with NLS curve fitting and B-spline smoothing, the accurate segmentation and extraction of the LV can be realized. Experiments show that the method can accurately and automatically identify and segment the LV in cardiac ultrasound images, and related indicators such as fps, Dice, MAD, and HD can reach 2.1–2.25 fps, 93.57 ± 1.97%, 2.57 ± 0.89 mm, and 6.68 ± 1.78 mm, respectively. Compared with other methods, the proposed method has a better segmentation accuracy and robustness. In particular, our method has a high computational speed, which is very important for real-time evaluation of cardiac function based on echocardiography. In addition, our method uses less training data to achieve better segmentation results. In short, our method can accurately segment LV ultrasound images, which is important for the accurate acquisition of clinical indicators for cardiac function evaluation, such as the EF, strain, and strain rate of the LV on echocardiography and will play a vital role in assisting doctors in clinical diagnosis.

## Figures and Tables

**Figure 1:** Block diagram of the proposed method.

**Figure 2:** Detection of LV based on YOLOv3.

**Figure 3:** Binarization results of LV endocardium images based on MRF: (a–d) the original frames extracted at the equal interval from the same echocardiogram and (e–h) the corresponding binarization results.

**Figure 4:** Fitting curve results of the LV subgraph in different sequences without and with constraints.

**Figure 5:** Extraction and segmentation of LV endocardium. (a) Result of binarization of the LV image using MRF model. (b) Morphological mask generated according to the fitted positioning curve. (c) Binary myocardial image obtained after mask processing. (d) Approximation result of the endocardium based on the three constraint points. (e) Result of smoothing the myocardium based on the B-spline method.

**Figure 6:** *P*‐*R* curve of the LV identification and constraint box based on the proposed method in this paper. (VS: ventriculus sinister; Lower left: the constraint point in the lower left corner; Lower right: the constraint point in the lower right corner; and Top: the constraint point on the top of the myocardial wall).

**Figure 7:** Binarization results of ultrasonic LV images using the Otsu method, *K*-means clustering method, and MRF model. The area enclosed by the blue line in (a) and (e) is the gold standard for the LV myocardium. (b, f) The binarization results obtained by using the Otsu method. (c, g) The binarization results obtained by using the *K*-means clustering algorithm. (d, h) The binarization results obtained by using the method proposed in this paper.

**Table 1:** Evaluation results of the YOLOv3-based LV and three bounding box positioning model using AP50.

	LV	Left_down	Right_down	Top
AP	100.00%	92.33%	95.44%	94.50%

**Table 2:** Comparison of binarization results obtained by different methods and gold standards.

	Otsu	*K*-means	MRF
Dice	0.58 ± 0.07	0.59 ± 0.06	0.88 ± 0.03

**Table 3:** Comparison of endocardial segmentation results by different methods.

Methods	Training set size (frame)	Computation speed (fps)	Dice (%)	MAD (mm)	HD (mm)
Hansson et al. [33]	0	0.3	—	2.58 ± 0.85	—
Qin et al. [34]	450	0.01	90.8 ± 1.7	2.0 ± 0.42	6.86 ± 1.71
Carneiro and Nascimento [35]	496	0.2	—	1.94 ± 0.51	—
The method without constraints	252	1.5–1.8	80.103 ± 2.13	7.06 ± 0.85	10.34 ± 3.51
*Proposed method*	252	2.1–2.25	93.578 ± 1.97	2.57 ± 0.89	6.68 ± 1.78

## Data Availability

The cardiac ultrasound imaging data used in this study were provided by the Ultrasound Imaging Department of the First Affiliated Hospital of Medical College of Shantou University, China, which is not open to the public because it would breach the privacy of the research.
